The article "Effects of hPMSCs on granulosa cell apoptosis and AMH expression and their role in the restoration of ovary function in premature ovarian failure mice" was retracted in 2022. Reasons: errors in the images; duplicated images; original data or images not available; unreliable data.

# Effects of hPMSCs on granulosa cell apoptosis and AMH expression and their role in the restoration of ovary function in premature ovarian failure mice

**DOI:** 10.1186/s13287-017-0745-5

**Published:** 2018-01-31

**Authors:** Hongqin Zhang, Qianqian Luo, Xueyan Lu, Na Yin, Dongli Zhou, Lianshuang Zhang, Wei Zhao, Dong Wang, Pengchao Du, Yun Hou, Yan Zhang, Wendan Yuan

**Affiliations:** 1 School of Basic Medical Sciences & Institute of Reproductive Diseases, Binzhou Medical University, Yantai, Shandong 264003 China; 2 School of Basic Medical Sciences, Binzhou Medical University, Yantai, 264003 China; 3 Health School of Laiyang, Laiyang, 265200 China; 4 State Key Laboratory of Stem Cell and Reproductive Biology, Institute of Zoology, Chinese Academy of Sciences, Beijing, 100101 China

**Keywords:** Placenta, Mesenchymal stem cell, Premature ovarian failure, Granulosa cells, Apoptosis, Anti-Müllerian hormone, Follicle stimulating hormone receptor

## Abstract

**Background:**

This study was performed to determine the effects of human placenta mesenchymal stem cell (hPMSC) transplantation on granulosa cell apoptosis and anti-Müllerian hormone (AMH) and follicle-stimulating hormone receptor (FSHR) expression in autoimmune drug-induced premature ovarian failure (POF) mice. The aim of this research is to investigate the mechanisms of hPMSCs on ovarian reserve capacity.

**Methods:**

The POF mice model was established by injection of zona pellucida 3 peptide (pZP3). hPMSC transplantation was conducted by intravenous injection into mice following pZP3 treatment. The follicle number was examined by histopathology. The serum levels of FSH, LH, E_2_, AMH and anti-zona pellucida antibody (AzpAb) were measured by enzyme-linked immunosorbent assay. AMH and FSHR expression in the ovary was analyzed by immunohistochemistry and western blot analysis. Granulosa cell apoptosis of the ovaries was examined by In Situ Cell Death Detection Kit. Granulosa cells were isolated and treated with SiAmh interference and hPMSC supernatant to observe the effects of AMH expression on granulosa cell apoptosis in vitro.

**Results:**

The results showed that hPMSC transplantation can significantly recover the estrus cycle in the POF group. Morphological staining showed that the basal follicles and sinus follicles after hPMSC transplantation were higher in POF mice than in those without treatment, and the follicle number was significantly decreased with atresia. The serum levels of FSH, LH and AzpAb in the hPMSC transplantation group were reduced considerably, but the E_2_ and AMH levels were significantly increased. After hPMSC transplantation, the AMH and FSHR expression in ovarian tissue was significantly higher than in the POF group as determined by immunochemistry and western blot analysis. The FSHR expression was shown in granulosa cells only, and FSHR expression increases with AMH expressed in the ovary; granulosa cell apoptosis was decreased following hPMSC transplantation. The same results were observed from the in-vitro study.

The article "Effects of hPMSCs on granulosa cell apoptosis and AMH expression and their role in the restoration of ovary function in premature ovarian failure mice" was retracted in 2022. Reasons: errors in the images; duplicated images; original data or images not available; unreliable data.

**Conclusions:**

hPMSC transplantation can significantly improve the serum levels of high gonadotropin and low estrogen of POF mice, promote follicular development, inhibit excessive follicular atresia and granulosa cell apoptosis, and improve the ovarian reserve capacity. The mechanism may be achieved by increasing the expression of AMH and FSHR in ovaries.

**Electronic supplementary material:**

The online version of this article (doi:10.1186/s13287-017-0745-5) contains supplementary material, which is available to authorized users.

## Background

Premature ovarian failure (POF) is a disease of ovarian dysfunction that seriously affects women’s physical and mental health, which refers to amenorrhea, ovarian atrophy, sexual hypoactivity and fertility decline after puberty of women and before the age of 40, and may lead to a series of syndromes of osteoporosis and cardiovascular disease [1–3]. The pathogenesis of this disease has not yet been understood fully. Ovarian failure is shown as a decline in ovarian reserve capacity [4]. Evaluation of ovarian reserve capacity in the clinic is of great importance for early detection of POF, prediction of fertility potential and menopause age. Reduced ovarian reserve is often referred to as a decreased number or quality of follicles and oocytes [5]. Folliculogenesis was related to anti-Müllerian hormone (AMH) expressed in the granulosa cells. AMH regulates the recruitment of follicles by limiting the number of oocytes recruited and growing follicles [6]. Therefore, AMH is emerging as a novel ovarian test marker involved in the pathogenesis of POF.

Currently, the prevention and treatment of POF are extremely difficult. The most commonly used hormone replacement therapy cannot effectively recover ovarian function [7]. Mesenchymal stem cells (MSCs) are the adult stem cells that have been studied in recent years and used to treat many diseases. MSCs can be isolated from a variety of tissues, especially human placenta. The human placenta-derived mesenchymal stem cells (hPMSCs) have gained wide attention due to their convenient isolation, less virus infection and low immunogenicity [8]. However, the application of hPMSC transplantation in the treatment of autoimmune ovarian injury and its effect on ovarian reserve capacity has not been investigated widely.

The article "Effects of hPMSCs on granulosa cell apoptosis and AMH expression and their role in the restoration of ovary function in premature ovarian failure mice" was retracted in 2022. Reasons: errors in the images; duplicated images; original data or images not available; unreliable data.

The study was performed on the POF mice model induced by zona pellucida glycoprotein 3 peptide (pZP3) injection. In this article, the effects of human placental mesenchymal stem cell therapy on ovarian reserve capacity, granulosa cells and related AMH and FSHR were studied. The data from this study suggested that hPMSCs provide a promising therapeutic method for patients with POF in the clinic.

## Methods

### Experimental animals and reagents

Female mice (Balb/c) aged 6–8 weeks were obtained from Ji'nan Pengyue Experimental Animal Breeding, Ltd (Shandong, China). Mice with a weight of 18–22 g were assigned randomly to the control group (*n* = 24), POF group (*n* = 24) or POF + hPMSCs group (*n* = 24). All animals were housed in the animal facility and were fed a standard pellet diet with free access to water. All of the experimental procedures were approved by the Institutional Animal Care and Use Committee at Binzhou Medical University. The study was conducted according to the National Research Council Guide for Care and Use of Laboratory Animals.

Zona pellucida glycoprotein 3 peptide (pZP3) was synthesized by an automatic peptide synthesizer (Zhongtai Biochemical Co. Ltd, Hangzhou, China), and 95% peptide purity was determined by HPLC analysis. The amino acid composition was checked by amino acid analysis and the amino acid sequence of the murine ZP330–342 peptides used in this study was NSSSSQFQIHGPR. The reagents used in the study include complete Freund’s adjuvant (CFA), Freund’s incomplete Adjuvant (FIA; *Mycobacterium tuberculosis* H37RA strain, 0.16 mg/mouse) (Sigma, USA), rabbit anti-mice FSHR antibody (Santa Cruz, USA) and the ELISA kit (Beijing Huaying Institute of Biological Technology).

### Establishment of the POF mice model

The pZP3-induced POF mice model was established according to the literature [9–11]. Each mouse was injected subcutaneously with 150 μl pZP3 at the foot, abdomen and back. After 2 weeks, pZP3 emulsified in FIA was injected subcutaneously. One week following the treatment of pZP3 with FIA, blood samples were collected by tail vein puncture. AZPAb was measured by ELISA in POF mice to confirm the successful injection of pZP3. In the control group, the expression of AZPAb was negative.

One week following the successful establishment of the POF model characterized by irregular estrous cycles, 1 × 10^6^ hPMSC cell suspension at the third generation was injected intravenously into mice through the tail vein according to a study published previously [12]. Two weeks after hPMSC transplantation, the blood and ovary tissue of POF + hPMSCs group mice were obtained for further experiment.

### Estrous cycle examination

Vaginal smear was performed under light microscopy. The type of estrous cycle was determined as shown by the proportions of nucleated and keratinized epithelial cells and leukocytes. The level of cycle abnormality (I–IV) was graded as follows: I, normal; II, regular cycles with a shortened estrus; III, irregular cycles with a prolonged diestrus and normal or prolonged estrus; IV, no cyclicity. Estrous cycle disorder is a distinguishing characteristic of ovarian function failure.

The article "Effects of hPMSCs on granulosa cell apoptosis and AMH expression and their role in the restoration of ovary function in premature ovarian failure mice" was retracted in 2022. Reasons: errors in the images; duplicated images; original data or images not available; unreliable data.

### Enzyme-linked immunosorbent assay

At the end of the study, blood samples were obtained from eyeball veins and centrifuged at 3220 ×g for 15 min. FSH, LH, E_2_, AMH and AzpAb levels in the serum were measured by ELISA kit (Lengton, Shanghai, China) according to the manufacturer’s instructions.

### Ovarian follicle counting and morphological analysis

At the end of the study, the mice were euthanized and ovaries were collected, which were fixed and stained with H&E for histopathology examination under light microscopy. Only the follicles containing an oocyte with a clearly visible nucleus were counted. Furthermore, the follicles were classified as primordial, primary, secondary and atresia follicle, according to the method described previously [13, 14]. Five slides were selected randomly in each group and five nonrepetitive views on each slide were selected for statistical analysis.

### Immunohistochemistry

The bilateral ovaries were fixed in the paraformaldehyde solution (4%), and then embedded in paraffin wax. The ovary tissues were sectioned at 4 μm. The slides were dewaxed in distilled water and incubated with the primary polyclonal rabbit antibodies of AMH and FSHR. The concentration of AMH and FSHR was 1:150 and antibodies were incubated for 12 hours at 4 °C in a humidity environment. Biotinylated secondary antibody anti-rabbit IgG was used on the sections for 1-hour incubation at 37 °C. Five sections on each slide were selected randomly for examination.

The German immunoreactive score criteria (IRS) were used to score the staining results. Briefly, staining signal intensity was graded as “0” (negative), “1” (weak), “2” (moderate) and “3” (strong); the extent of staining cells was graded as “0” (<5%), “1” (5–25%), “2” (25–50%), “3” (50–75%) or “4” (> 75%). Values of staining intensity and staining extent were multiplied as a final IR score [15].

### Western blot analysis

The mice were anesthetized and bilateral ovaries were collected. The tissue homogenates were centrifuged at 12,000 × *g* at 4 °C for 10 min. Bradford’s method was used to measure the protein concentration of supernatants [16]. The total proteins were subjected to electrophoresis in 8% SDS-PAGE gels and transferred onto a PVDF membrane. Subsequently, membranes were probed overnight at 4 °C with anti-FSHR (1:100), anti-AMH (1:1000) and anti-GAPDH (1:800; Goodhere, China) polyclonal antibodies. At room temperature, the horseradish peroxidase-conjugated secondary antibody (1:5000) was incubated on the membrane for 1 hour. The ECL Plus western blot detection system (Thermo Scientific) was used to detect the immunoreactive signals.

The article "Effects of hPMSCs on granulosa cell apoptosis and AMH expression and their role in the restoration of ovary function in premature ovarian failure mice" was retracted in 2022. Reasons: errors in the images; duplicated images; original data or images not available; unreliable data.

### In-situ cell death detection

Apoptosis in the granulosa cells was examined by the In Situ Cell Death Detection Kit (Roche, USA) on the basis of the manufacturer’s instructions. DAPI was used to stain the nucleus, and the staining signals of apoptosis were evaluated using fluorescence microscopy (Leica, Germany). Additional tissue sections were added for the negative and positive labeling controls.

### Isolation and culture of hPMSCs

The use of human placenta tissue was approved by the Institutional Ethics Committee. hPMSCs were isolated and cultured according to Chen [8]. The specific contents were attached to the (Additional file 1). The membrane and intracytoplasmic molecular markers of hPMSCs were examined using flow cytometry (FCM) to confirm the phenotype of the cells [8].

### Isolation, culture and identification of granulosa cells

The Balb/c mice in the control group were administered 20 U PMSG (5000 U/5 ml). After 48 hours, the ovaries were collected and granulosa cells were isolated mechanically according to a previous study [17]. The culture solution contains DMEM medium 1× (1:1) with 10% FBS, FSH 100 U and 1% antibiotic, and the granulosa cells were incubated at 37 °C with 5% CO_2_ for 48 hours. After incubation, cell numbers were determined using a hemocytometer at a concentration of 10,000 cells per well in a culture plate. The medium was then removed using a pipette and washed with PBS. The plates were incubated with the primary polyclonal rabbit antibodies:anti-FSHR (1:150) for 12 hours at 4 °C in a humidity chamber. Biotinylated secondary antibody anti-rabbit IgG (Dylight 549, 1:300) was applied to the sections for 30-min incubation at 37 °C. After DAPI transfused the nucleus, the signals from each staining were examined by fluorescence microscopy.

### SiAmh interference and hPMSC supernatant treatment

For examining the effects of AMH on granulosa cell apoptosis, treatment was conducted using SiAmh interference for 24 hours. The SiAmh interference study was performed according to the kit instruction when the cell growth reached about 80%. After interference, regular culture medium was replaced 6–8 hours later and cells were cultured for 48 hours. The SiAmh + hPMSCs groups were added to the culture medium which mixed with the hPMSC supernatant at a ratio of 1:1. After 48-hour cell transfection, total RNA was extracted using the Trizol method. After reverse transcription, PCR was used to determine the expression of AMH mRNA in the granulosa cells. Total RNA (1 μg) was applied to the reverse transcription. The reaction condition was as follows: 10 min at 65 °C (pre denaturation), 60 min at 50 °C (initial denaturation), 5 min at 85 °C (amplification). PCR amplification was performed according to the steps of Roche fast start universal SYBR Green master (ROX). The primer sequences are as follows: AMH-F, 5′-TGCTAGTCCTACATCTGGCTGA-3′; and AMH-R, 5′-GTCCAGGGTATAGCACTAACAGG-3′.

The article "Effects of hPMSCs on granulosa cell apoptosis and AMH expression and their role in the restoration of ovary function in premature ovarian failure mice" was retracted in 2022. Reasons: errors in the images; duplicated images; original data or images not available; unreliable data.

Cell apoptosis was detected by flow cytometry. After 48-hour cell transfection, the cells were collected and digested with pancreatic enzymes and washed twice with cold PBS. Then 500 ml Annexin V Binding Buffer cell suspension, 5 μl FITC Annexin V and 5 μl PI were added. The cells were then cultured at room temperature for 15 min for flow cytometry analysis within 1 hour.

### Data analysis

Statistics were expressed using the mean ± SEM and analyses were performed with SPSS 13.0 software. One-way analysis of variance (ANOVA) was used between the three groups and statistically significant difference was expressed as *P* < 0.05.

## Results

### General status and body weight change of mice

There was no significant weight change among the three groups before pZP3 treatment. Following pZP3 treatment, a statistically considerable difference between the three groups was observed (*P* < 0.01), as shown in Fig. 1a. There was a significant weight loss in the POF group compared to the control and hPMSC groups. The average weight of mice in the POF group was 21.71 ± 0.96 g as compared to 23.38 ± 1.41 g in the control group.

**Fig. 1:** **a** Body weight (g) and **b** ovary weight (g) of the three groups before and after pZP3 treatment compared at the same time. **P < 0.01. hPMSC human placenta mesenchymal stem cell, POF premature ovarian failure

### hPMSC phenotype characterization

Cells isolated from human placenta began to form individual colonies after 7–10 days of inoculation. The morphology of cells appears similar to the fibroblasts, as shown in Fig. 2b. These adherent cells can be passaged easily by multiple trypsinization. A homogeneous cell population was observed after three passages. Even following 10 passages, the cells still retain normal morphology. The phenotype analysis by immunofluorescence showed that the cells express positive mesenchymal progenitor markers with CD73, CD90 and CD105. The hematopoietic cell surface markers CD14, CD34 CD19 and HLA-DR are shown negative (Fig. 2a). In an ex-vivo conditional culture system, hPMSCs can be induced to develop into different lineages. In osteoblastic induction medium, von Kossa staining showed that calcium was deposited in the cells (Fig. 2c). In adipogenic induction medium, fat globules were present in the cytoplasm, and Oil Red O staining was positive (Fig. 2d). The results of this part were in conformity with the previous literature report on the confirmation of hPMSC phenotype characterization [8].

The article "Effects of hPMSCs on granulosa cell apoptosis and AMH expression and their role in the restoration of ovary function in premature ovarian failure mice" was retracted in 2022. Reasons: errors in the images; duplicated images; original data or images not available; unreliable data.

**Fig. 2:** Confirmation of hPMSC characteristics by cell surface marker staining and differentiation capability of cells. Surface markers of hPMSCs measured by flow cytometry. **a** Green line in each histogram represents isotype control staining; specific expression of indicated cell surface marker presented as blue histograms. **b**–**d** Cells cultured under various conditions to differentiate to osteoblast or adipogenesis cells. **b** Normal hPMSCs show fibroblast-like morphology. **c** Osteoblasts confirmed by Alizarin Red staining; dark red staining shows calcium deposition. **d** Adipogenesis confirmed by accumulation of neutral lipid vacuoles inside cells with Oil Red O stain. Scale bar: 200 μm. Magnification × 200

### Effects of hPMSC transplantation on estrous cycles

The estrous cycles were examined over a 5-week period following pZP3 treatment. Regular estrous cycles in the control group were shown in 86.96% of mice and lasted 4–6 days, which includes proestrus for 1 day, estrus for 1–2 days, metestrus for 1 day and diestrus for 1–2 days (Fig. 3a–d). However, the significantly irregular estrous cycles were observed in POF mice as shown in Fig. 3e, f. Only 14.29% of mice showed a regular cycle in the POF group. However, following hPMSC transplantation, 62.5% of mice in the POF group showed a regular estrous cycle. The normal estrous cycles were significantly higher as compared to POF mice (*P* < 0.01). The results indicated that following pZP3 treatment, ovarian function was injured and the POF mice model was established successfully due to ovarian injury. After hPMSC transplantation, ovarian function has been significantly improved as seen in the increase of the normal estrous cycle.

**Fig. 3:** Effects of hPMSC transplantation on estrous cycles for pZP3-induced POF mice. Normal estrous cycles: **a** proestrus, **b** estrus, **c** metestrus, **d** diestrus. **e** Four patterns of estrous cycles were graded with the severity of abnormality (I–IV) as follows: I, normal; II, regular cycles with a shortened estrus; III, irregular cycles with a prolonged diestrus and normal or prolonged estrus; IV, no cyclicity. *y* axis represents the cycle day in proestrus or estrus (p-e) and metestrus or diestrus (m-d). Each circle (○) represents one mouse. Illustration is only represented by a mouse and the main purpose is to show the change of estrus cycle. **f** Total numbers of mice from each group categorized into the various estrous patterns (I–IV). **P < 0.01 indicates the statistically significant difference of the estrous cycle in mice with and without hPMSC transplantation. Data presented as mean ± SD (*n* = 24). hPMSC human placenta mesenchymal stem cell, POF premature ovarian failure

The article "Effects of hPMSCs on granulosa cell apoptosis and AMH expression and their role in the restoration of ovary function in premature ovarian failure mice" was retracted in 2022. Reasons: errors in the images; duplicated images; original data or images not available; unreliable data.

### The serum of FSH, E_2_, LH, AMH and AzpAb levels

As shown in Fig. 4, following pZP3 treatment the serum gonadotropin including FSH and LH and AZPAb levels in POF mice were higher but E_2_ and AMH levels were lower than the control group. Statistically significant difference between two groups at the same time was expressed as *P* < 0.01. Compared with the POF group, the serum E_2_ and AMH levels were increased but gonadotropin and AZPAb levels were decreased after hPMSC transplantation (*P* < 0.001).

**Fig. 4:** Effects of pZP3 treatment on serum **a** E_2_, **b** FSH, **c** LH, **d** AMH and **e** AzpAb Concentration in mice with or without hPMSC transplantation. Values expressed as mean ± SEM (*n* = 24). **P < 0.01, ***P < 0.001 indicate the statistically significant difference between the groups. E_2_ estradiol, FSH follicle stimulating hormone, LH luteinizing hormone, AMH anti-Müllerian hormone, AzpAb anti-zona pellucida antibodies, hPMSC human placenta mesenchymal stem cell, POF premature ovarian failure

### Histological examination and follicle count

Most healthy follicles, including primordial follicles, primary follicles, secondary follicles and atretic follicles, were observed in the ovaries of the control group (Fig. 5a). In contrast, the ovaries of pZP3 immunization mice were withered with most mesenchymal cells in a fibrous matrix. The number of follicles was counted at every stage (atretic or normal follicles) among the three groups. The numbers of follicles at any stage were decreased compared to the control group. Granulosa cells were arranged irregularly and lymphocyte infiltration was observed among the follicles (Fig. 5b). The morphological changes of the hPMSC treatment group were better than the POF group (Fig. 5c). The results showed a considerably lower number of atretic follicles but more normal follicles in the ovaries of the hPMSC transplantation group than in the POF group.

**Fig. 5:** Histopathological examination and follicle counts in ovaries. **a** Control group. **b** POF group. **c** hPMSC treatment group. **d** Summary of follicle count from the ovaries of each group. The following different types of ovarian follicles were observed: primordial follicle (▲), primary follicle (▼), secondary follicle (■), atretic follicle (●). Magnification × 100. Scale bar: 200 μm. Data presented as mean ± SD. *P < 0.05, ***P < 0.001 indicates the statistically significant difference between the groups with and without pZP3 treatment. hPMSC human placenta mesenchymal stem cell, POF premature ovarian failure

The article "Effects of hPMSCs on granulosa cell apoptosis and AMH expression and their role in the restoration of ovary function in premature ovarian failure mice" was retracted in 2022. Reasons: errors in the images; duplicated images; original data or images not available; unreliable data.

### Expression of AMH and FSHR

Expression of AMH and FSHR was detected by immunohistochemical analysis. It was noted that most atretic follicles can be observed. The data showed that the expression of AMH and FSHR was decreased in ovaries of pZP3-induced POF mice compared to the control group (*P* < 0.05). The positive cells for AMH mainly occurred in the preantral and small antral follicles. In comparison, the majority of healthy follicles were observed in the ovaries from the POF + hPMSCs group, with a significantly increased secretion of AMH and FSHR (Fig. 6d, h).

**Fig. 6:** Effects of hPMSC transplantation on AMH and FSHR expression in ovarian tissues by immunochemistry analysis. Cells with **a–d** FSHR and **e–h** AMH expression shown brown in the cytoplasm. Cell nucleus stained blue. Data expressed as mean ± SD. Statistical differences between the groups: *P < 0.05, **P < 0.01, ***P < 0.001. Scale bar: 50 μm. Magnification × 400. FSHR follicle stimulating hormone receptor, AMH anti-Müllerian hormone, hPMSC human placenta mesenchymal stem cell, POF premature ovarian failure

Furthermore, the protein expression of AMH and FSHR in the ovaries was measured by western blot analysis. The data showed that AMH and FSHR expression in the ovarian tissues of the POF group was decreased extensively compared to the control group. After hPMSC treatment, AMH and FSHR expression was significantly increased in the POF group as revealed in Fig. 7.

**Fig. 7:** AMH and FSHR expression in the ovaries by western blot analysis. **a** Representative image of western blot analysis. Quantization on **b** FSHR and **c** AMH protein expression. The housekeeping gene was GAPDH used to quantitate protein expression. ImageJ software used to quantitate the intensity of AMH and FSHR. *P < 0.05, **P < 0.01 indicates significant differences among three groups. Data expressed as mean ± SEM. FSHR follicle stimulating hormone receptor, AMH anti-Müllerian hormone, hPMSC human placenta mesenchymal stem cell, POF premature ovarian failure

### Granulosa cell apoptosis

Apoptosis of granulosa cells is close to the development of follicular atresia. The results revealed that the number of apoptotic cells in the POF group was significantly increased compared to the control group (Fig. 8). However, after treatment with hPMSCs, the apoptosis numbers of granulosa cells were significantly decreased. The data suggest that apoptosis of granulosa cells plays an important role in the development of ovarian function failure in POF mice. hPMSC implantation could inhibit cell apoptosis to recover ovarian function.

The article "Effects of hPMSCs on granulosa cell apoptosis and AMH expression and their role in the restoration of ovary function in premature ovarian failure mice" was retracted in 2022. Reasons: errors in the images; duplicated images; original data or images not available; unreliable data.

**Fig. 8:** Apoptosis of granulosa cells in ovarian tissues measured by TUNEL analysis. Apoptotic cells shown as green fluorescence with FITC staining. The nucleus was stained with DAPI, shown as blue fluorescence. Magnification × 400. DAPI 4′,6-diamidino-2-phenylindole, hPMSC human placenta mesenchymal stem cell, POF premature ovarian failure

### Granulosa cell culture and identification

The granulosa cells were isolated from ovarian tissues. Cell morphology is shown in Fig. 9. The morphology of the granulosa cells was round and the cells were adherent after 24 hours, exhibiting polygonal and fiber-like structures. After follicle-stimulating hormone receptor (FSHR) immunostaining, GCs were stained red with Dylight 549, which accounted for approximately 80–85% of the adherent cells. The cells stained with Dylight 549 were the GCs, indicating that GCs derived from mice were successfully cultured in vitro.

**Fig. 9:** Morphological changes of granulosa cell culture. FSHR expression in cells under fluorescent microscope. blue, DAPI. red, Dylight 549. Scale bar: 50 μm. Magnification × 400. DAPI 4′,6-diamidino-2-phenylindole

### SiAmh interference and hPMSC supernatant on apoptosis

To further clarify the effects of AMH and supernatant of hPMSCs on granulosa cell apoptosis, SiAmh interference was involved in the granulosa cell culture and apoptosis of granulosa cells was detected. Compared with the control group, the Amh mRNA level was significantly decreased in SiAmh groups as shown in Fig. 10a. After staining with Annexin V-FITC and PI in granulosa cells, the apoptotic cells were counted by flow cytometry. Apoptosis cells are shown at the late stage (*x* axis) and the early stage (*y* axis). The percentage of apoptotic granulosa cells (shown in Fig. 10c–e) are 13.35 ± 1.25% in the control group, 30.63 ± 1.21% in the SiAmh group and 23.51 ± 1.67% in the SiAmh + CM group, respectively. The apoptosis rate in the SiAmh group was significantly higher than in the control group (*P* < 0.01). However, the apoptosis rate of granulosa cells was significantly decreased following supernatant of hPMSC treatment (*P* <0.01).

**Fig. 10:** Relative Amh mRNA expression after SiAmh interference and the apoptosis rate of granulosa cells measured by flow cytometry. **a** Relative level of Amh mRNA in granulosa cells after transfection of siAmh. *P < 0.05. **b** Comparison of percentage of apoptotic cells in the three groups. **P < 0.01. Apoptosis percentage of granulosa cells in the **c** control group, **d** SiAmh group and **e** SiAmh + CM group. SiAmh? small interfering Amh; CM: conditioned medium

The article "Effects of hPMSCs on granulosa cell apoptosis and AMH expression and their role in the restoration of ovary function in premature ovarian failure mice" was retracted in 2022. Reasons: errors in the images; duplicated images; original data or images not available; unreliable data.

## Discussion

POF, 1–3% of adult women being affected [2], has a profound impact on physical and mental health. At present, hormone replacement therapy (HRT) has been applied in the clinic to treat patients with POF [7]. However, HRT not only has noticeable side effects, but also could increase the risk of gynecological tumors with long-term application. Moreover, HRT neither inhibits the continuous rise of FSH nor fundamentally repairs the impaired ovarian function. In recent years, much more attention had been paid to research into mesenchymal stem cells (MSCs) for repair after injury. The research has shown that MSCs were located in the amniotic fluid, amniotic membrane and umbilical cord and demonstrated some protective effects on POF ovarian injury caused by chemotherapy [18–20]. Additionally, human placenta mesenchymal stem cells (hPMSCs) have become widely used in research because of their abundant source, easy collection, culture in vitro, convenient induction and expansion, low immunogenicity, no oncogenicity and ethical restriction [8]. Also, hPMSCs were regulated by estrogen and progesterone because of progesterone receptor and estrogen receptor alpha expression under physiological conditions [21]. In the current study, the cultured hPMSCs were injected into the POF mice via the tail vein to investigate their role and mechanisms in the treatment of POF. The results showed that the atretic follicle number significantly reduced but mature follicles increased, while follicles at all levels began to appear after hPMSC transplantation. The granulosa cells in the ovary increased considerably. In comparison, apoptosis cells are dramatically decreased in the hPMSC transplantation group compared to the control group. To assess an individual’s ovarian reserve, FSH and estradiol (E_2_) levels in the serum at the early follicular phase have been measured. In our study, the serum levels of FSH and LH in the hPMSC transplantation group were reduced, but the E_2_ level was increased. These statistics imply that hPMSC transplantation plays a vital role in the recovery of ovarian function in POF mice.

The regulation of follicular development was mainly affected by the local cytokines of the ovary, and the interactions between the granulosa cells and the oocytes played an important role in regulation [22–24]. AMH is one factor of the transforming growth factor beta (TGF-β) superfamily. AMH had a particular inhibitory effect on follicular development and primordial follicle recruitment. It also participates in selection of the dominant follicles and plays an important role in follicle growth [25, 26]. It had been shown that the TGF-β/Smad signaling pathway is an essential way to regulate follicular development [27, 28]. AMH is expressed in granulosa cells rather than membrane cells, oocytes and ovarian stromal cells. It has greatest expression in granulosa cells of preantral and small antral follicles (diameter < 4 mm). There is almost no AMH expression in the antral follicles with a diameter of 4–8 mm [29–31]. In addition, there will be no AMH expression when follicles become atretic.

The article "Effects of hPMSCs on granulosa cell apoptosis and AMH expression and their role in the restoration of ovary function in premature ovarian failure mice" was retracted in 2022. Reasons: errors in the images; duplicated images; original data or images not available; unreliable data.

In our study, the data showed that AMH was expressed in the antral and preantral follicles by immunohistochemical analysis. The serum AMH level was basically consistent with the quantitative analysis of AMH in the ovaries by immunohistochemistry and western blot analysis. The study conducted by Ingraham et al. [32] showed that AMH receptor was expressed only in the gonads and that AMH played a role in follicular development in a paracrine or autocrine manner. Also, studies have shown that the level of AMH in serum is closely related to the number of primordial follicles and growing follicles. The number of ovarian primordial follicles in the POF mouse model decreased, which may be due to the fact that the decreased level of AMH in serum increased the number of primordial follicles becoming the growing follicles, and decreased the number of the primordial follicles, resulting in premature depletion of the primordial follicle pool.

As reported, the follicles become atretic when 10% of granulosa cells have undergone apoptosis [33]. This indicates that granulosa cell apoptosis plays a vital role in the development of follicular atresia. Our study showed that the number of apoptotic granulosa cells and atretic follicles in POF mice was significantly increased compared to the control mice. However, the apoptotic granulosa cells and atretic follicles were decreased after the hPMSC treatment, while other types of follicles appeared in the ovaries, which suggested that hPMSCs may act on AMH expression through the cytokines secreted from granulosa cells. In addition, our study showed that the protein expression of FSHR in the ovaries of POF mice significantly increased, but decreased after hPMSC treatment. Inhibition of FSHR expression in POF mice following hPMSC treatment may be mediated by AMH. This is consistent with the report that AMH can reduce FSHR mRNA levels in human granulosa cells [24].

To further clarify the role of hPMSCs in improving the ovarian reserve via mediating granulosa cell apoptosis and AMH expression, we conducted the study by culturing granulosa cells with SiAmh interference. Since FSHR was only expressed in granulosa cells, the immunofluorescence method was used to confirm the cell type of granulosa cells in culture. The results of SiAmh interference and PCR analysis showed that AMH expression was significantly reduced but apoptosis granulosa cells were increased. The data suggest that AMH was involved in granulosa cell apoptosis. When granulosa cells were incubated with hPMSC supernatant after SiAmh interference, granulosa cell apoptosis was significantly reduced. This suggested that cytokines secreted by hPMSCs may be involved in the inhibition of granulosa cell apoptosis due to Amh mutation. The results from the in-vitro study support the results obtained from the in-vivo study. This further demonstrates that hPMSCs could reduce granulosa cell apoptosis and then enhance the ovarian reserve capacity via regulating AMH secretion and inhibiting granulosa cell apoptosis.

The article "Effects of hPMSCs on granulosa cell apoptosis and AMH expression and their role in the restoration of ovary function in premature ovarian failure mice" was retracted in 2022. Reasons: errors in the images; duplicated images; original data or images not available; unreliable data.

In summary, hPMSC transplantation can obviously improve the state of the serum levels of high gonadotropin and low estrogen of POF mice, promote follicular development, inhibit excessive follicular atresia and granular cell apoptosis, and improve the ovarian reserve capacity. These data demonstrate that the mechanisms of hPMSC transplantation promote ovarian function.

## Conclusions

hPMSC transplantation could recover ovarian function through inhibition of granulosa cell apoptosis and follicular atresia by upregulation of AMH and FSHR expression of granulosa cells in POF mice. It has the potential to provide a promising therapeutic method for patients with POF in the clinic.

## Additional file

Additional file 1: Presents isolation and culture of hPMSCs (DOCX 12 kb)

## Abbreviations

AMH: Anti-Müllerian hormone
ANOVA: One-way analysis of variance
AzpAb: Anti-zona pellucida antibody
CFA: Complete Freund’s adjuvant
DMEM: Dulbecco’s modified Eagle’s Medium
E_2_: Estradiol
ELISA: Enzyme-linked immunosorbent assay
FCM: Flow cytometry
FIA: Freund’s incomplete adjuvant
FSH: Follicle stimulating hormone
FSHR: Follicle stimulating hormone receptor
GC: Granulosa cell
hPMSC: Human placenta mesenchymal stem cell
LH: Luteinizing hormone
MSC: Mesenchymal stem cell
POF: Premature ovarian failure
pZP3: Zona pellucida 3 peptide
TGF-β: Transforming growth factor beta
